# Antibodies against Hsp60 and Hsp65 in the sera of women with ovarian cancer

**DOI:** 10.1186/1757-2215-7-30

**Published:** 2014-03-11

**Authors:** Piotr Bodzek, Robert Partyka, Aleksandra Damasiewicz-Bodzek

**Affiliations:** 1 Department of Gynaecology, Obstetrics and Oncological Gynaecology, Medical University of Silesia, Batorego 15, 41-902 Bytom, Poland; 2 Department of Chemistry, Medical University of Silesia, Zabrze, Poland; 3 Department of Anesthesiology, Intensive Treatment and Emergency Medicine, Medical University of Silesia, Katowice, Poland

**Keywords:** Anti-Hsp60 and anti-Hsp65 in ovarian cancer

## Abstract

**Background:**

The aim of this study was to evaluate the concentrations of IgG antibodies against Hsp60 and Hsp65 in sera of patients with ovarian cancer at various stages of clinical progress and for different histopathological types of disease.

**Methods:**

Serum samples from 149 patients with ovarian carcinoma and 80 healthy women were investigated. The concentrations of anti-Hsp60 and anti-Hsp65 antibodies were determined using the enzyme-linked immunosorbent assay technique.

**Results:**

The mean concentrations of anti-Hsp60 and anti-Hsp65 antibodies in the patients with ovarian cancer did not differ significantly from the mean levels in healthy women. Analysis in relation to the clinical progression stage showed that the concentrations of these antibodies were higher when the neoplastic process was less advanced and at early stages significantly higher than in control group. Mean concentrations of both antibodies were not significantly different in relation to the histological type of the ovarian cancer. The use of chemotherapy as a primary anticancer treatment did not cause a significant change in the concentration of anti-Hsp60 antibodies, but the mean level of anti-Hsp65 after this treatment was significantly higher than in control group.

**Conclusions:**

The immunological response to Hsp60/65 is increased in early clinical stages of ovarian cancer and the level of anti-hsp60/65 antibodies may be then a helpful diagnostic marker. Even antibodies against highly homologous Hsps may be cross-reactive only partially and differ by some functional properties.

## Background

Ovarian cancer is a frequent cause of death in women in highly developed countries. This is caused, on one hand, by too late diagnosis (no early clinical symptoms, no specific diagnostic markers), and on the other – by therapeutic problems, particularly at the late stage of disease. Most patients with advanced ovarian cancer respond well to initial chemotherapy, however, within two years chemoresistant recurrence follows.

In recent years considerable attention has been paid to the important role of heat shock proteins (Hsps) in various carcinogenesis processes and their participation in developing resistance to anticancer treatment [1]. Hsps are excessively expressed in numerous malignant neoplasms in humans, including genital cancers. They participate in tumour cells proliferation, their differentiation, invasion, metastasis, death and recognition by the immune system [2,3]. There is evidence that some Hsps, on one hand, protect cells against apoptosis inducing factors, like cytokines, ionising radiation or oxidative stress [4,5], while on the other, excessive expression of these proteins induced by chronic cell stress may result in apoptosis inhibition and thus facilitate cell neoplastic transformation [3,5]. Moreover, chaperone molecules may then protect transformed neoplastic cells, renaturating their cell proteins damaged by cytostatic agents used in anticancer therapy (chemo- or radiotherapy), thus contributing to increased aggressiveness of neoplasm and its resistance to treatment (2).

The role of some Hsp in processes of cancerogenesis, including ovarian cancer, has been considerably well described. However, still little is known about a possible role of a protein of 60 kDa – Hsp60. Hsp60 is an evolutionary highly conserved protein, which analogues in prokaryotic cells include mycobacterial Hsp65. In most cells, human Hsp60 is present constitutively in mitochondria, where it plays a role in protein assembly, folding and transport [1]. In conditions stressful to a cell, however, not only changes in its intracellular distribution may occur, but also it may be expressed on a cell surface or released to the intercellular space, indicating a possible role of that protein as an intercellular signalling molecule. It also exhibits immunoregulatory properties by inducing a proinflammatory response in cells responsible for the innate immune response, like macrophages, dendritic cells or endothelial cells [6].

Extracellular forms of heat shock proteins, including Hsp60, also behave as autoantigens and induce host’s B- and T-cell immune response. Anti-Hsps antibodies can be found in healthy people and they can be treated as a part of the natural autoantibodies spectrum [7,8]. Their increased number can then reflect increased extracellular expression of shock proteins, caused by cells’ specific pathologic conditions or their modified activity [7]. Anti-Hsps immunization may also be caused by heterologous Hsps, e.g. of bacterial origin, as some bacterial heat shock proteins, like Hsp65, are also surface antigens, against which antibodies are produced in the immune response process [9]. Considering their high inter-species conservatism, the immune response to heterologous Hsps may also be a source of cross-reactivity with autoantigens [9,10]. Increased levels of anti-Hsps antibodies have already been observed in many diseases, particularly resulting from autoagression (review in 7). It was also demonstrated that levels of circulating Hsps and anti-Hsps antibodies could be useful biomarkers for carcinogenesis in some tissues, as well as prognosis factors for survival and susceptibility to treatment [2,7].

Presence of Hsp60 and anti-Hsp60/65 antibodies in serum of patients with ovarian cancer, however, still remains a new research field, and studies conducted so far often gave contradictory results. The aim of this study was, therefore, to evaluate levels of IgG antibodies against these proteins in serum of patients with ovarian cancer at different stages of clinical progress and with various histopathological types of disease.

## Material and methods

The study included 149 women with ovarian cancer, hospitalised at the Department of Gynaecology, Obstetrics and Oncological Gynaecology of Medical University of Silesia in Bytom. Patients with co-occurring diseases, such as diabetes, advanced atherosclerosis, hypertension, etc., were excluded from the study. The control group consisted of 80 healthy women without any history of cancer.

The blood samples (about 5 ml in volume) were obtained at 8.00 a.m., in the fasted state, from antecubital veins and they were centrifuged immediately. The collected sera had been stored at -70°C until assays could be performed.

The study protocol was approved by the Local Bioethics Commission of the Medical University of Silesia in Katowice. All women included were informed about the aim of the study and gave their written consent for participation.

The concentrations of IgG antibodies against Hsp60 (anti-Hsp60) and Hsp65 (anti-Hsp65) in studied serum samples were determined with the enzyme-linked immunosorbent assay (ELISA). The antigens used were recombinant human Hsp60 (Enzo Life Sciences Inc., Farmingdale, NY) and recombinant Hsp65 from Mycobacterium bovis (Calbiochem, San Diego, CA). The ELISA plates (Maxisorp, Nunc, Denmark) were coated with antigen solution at a concentration 2 mg/ml of 50 mM carbonate buffer at pH = 9.6. Studied sera were diluted 400× (optimal dilution was chosen experimentally) in 0.5% bovine serum albumin in phosphate buffered saline with Tween-20. Calibration was performed using pooled sera from about 100 of the healthy blood donors. The 400× dilution was assumed to correspond to 100 arbitral units/ml (AU/ml). A calibration curve consisted of 6 standards, with levels from 0 to 400 AU/ml. Incubation with studied sera and standards was conducted for 24 hours at 4°C. For detection of bound IgG antibodies, a goat anti-human IgG antibody conjugated with a horseradish peroxidase (Sigma, St. Louis, MO) was used. A tetramethylbenzidine solution (Sigma, St. Louis, MO) was used as a substrate for an enzymatic reaction. Absorbances were read with the Power Wave XS plate reader (BioTek, Winooski, VT) at 450 nm (reference wavelength - 630 nm), and results were processed with the KCJunior software (BioTek, Winooski, VT). The intra-assay variation was 8%. Determinations were done during one series. The assay sensitivity was about 1 AU.

The obtained results were presented using basic descriptive statistics parameters. The accordance of the data distribution with the normal distribution was checked with the Szapiro-Wilk test. The groups were compared using non-parametric Kolmogorov-Smirnov and *U* Mann–Whitney tests, and the test of differences between structure indications. For study of variability in the group of patients with ovarian cancer, the Kruskal-Wallis ANOVA rank test was used. Correlations between parameters were assessed with the Spearmann’s rank correlation test. The significance level of p < 0.05 was considered to be statistically significant. Calculations were conducted with the application STATISTICA for Windows, version 10.0, from StatSoft Inc. (Tulsa, OK).

## Results

The mean age (56.2 ± 10.5 years) of studied women with ovarian cancer was comparable to the age (52.8 ± 8.2 years) of women in the control group (p > 0.05). Of 149 studied patients, in 72 patients ovarian cancer was diagnosed for the first time and they were not treated yet, while 77 patients already underwent previous anticancer chemotherapy. The studied group included patients with various histopathological forms of ovarian cancer and at different clinical stages. Their detailed characteristics are presented in Table 1.

**Table 1:** Clinical characteristics of examined women with ovarian cancer (n = 149)

**Clinical data**	**Number of patients (%)**
**Antineoplastic treatment:**	
• Untreated so far	72 (48,3)
• After chemotherapy	77 (51,7)
**Histopathological type of ovarian cancer:**	
• *Adenocarcinoma papillare serosum*	82 (55,0)
• *Adenocarcinoma mucinosum*	44 (29,6)
• *Adenocarcinoma endometrioides*	23 (15,4)
**Stage of the clinical progresion (by FIGO):**	
• I	25 (16,8)
• II	31 (20,8)
• III	60 (40,3)
• IV	33 (22,1)

The mean concentrations of anti-Hsp60 and anti-Hsp65 antibodies in the whole group of patients with ovarian cancer did not differ significantly from the mean levels of these antibodies in the control group of healthy women (Table 2). Positive results (values exceeding 90^th^ percentile for the control group) were observed in 21.8% patients with ovarian cancer for anti-Hsp60 levels and in 20.6% patients for anti-Hsp65 levels. In both cases, the percentage of values considered to be positive was significantly higher than in the control group.

**Table 2:** Concentrations of anti-Hsp60 and anti-Hsp65 IgG antibodies in group of women with ovarian cancer and in control group

	**Ovarian cancer**	**Controls**
	**n = 149**	**n = 80**
**Anti-Hsp60** (AU/ml)	93,91 ± 127,75	62,42 ± 33,92
(mean ± SD)		
**% of positive resullts**	21,8%*	10%
(> 90 percentile for control group)	p = 0.024	
**Anti-Hsp65** (AU/ml)	97,06 ± 169,95	56,35 ± 35,58
(mean ± SD)		
** % of positive resullts**	20,6%*	10%
(> 90 percentile for control group)	p = 0,039	

*p < 0.05 in group of women with ovarian cancer compared to control group.

The analysis depending on the disease clinical stage (FIGO) showed that the mean levels of anti-Hsp60 and anti-Hsp65 antibodies were higher when the neoplastic process was less advanced (Table 3). The mean concentrations of both antibodies in patients at the I and the II clinical stage are significantly higher than in the control group. The mean levels of both antibodies in patients at the I stage are significantly higher than at the III and the IV stages, and mean levels at the II stage are significantly higher than at the IV stage. The similar observations were done for the percentages of positive values (details in Table 3).

**Table 3:** Concentrations of anti-Hsp60 and anti-Hsp65 IgG antibodies in group of women with ovarian cancer depending on stage of clinical disease progression (by FIGO) and in control group

	**Stage of clinical disease progression (by FIGO)**				**Controls**
	**I**	**II**	**III**	**IV**	**n = 80**
	**n = 25**	**n = 31**	**n = 60**	**n = 33**	
**Anti-Hsp60** (AU/ml)	126,99^a)b)e)^	97,15^c)e)^	91,92	70,87	62,42
(mean ± SD)	± 121,90	± 91,82	± 160,11	± 78,70	± 33,92
** % of positive results**	46%^f)^	27%^f)^	17%	17%	10%
(> 90 percentile for control group)	p = 0.0000	p = 0.0213	p = 0.2047	p = 0.2861	
**Anti-Hsp65** (AU/ml)	190,34^a)b)e)^	97,80^c)e)^	89,36^d)^	44,17	56,35
(mean ± SD)	± 337,27	± 90,59	± 137,58	± 26,07	± 35,58
** % of positive results**	46%^f)^	27%^f)^	21%	0%^f)^	10%
(> 90 percentile for control group)	p = 0.0000	p = 0.0213	p = 0.0594	p = 0.0493	

^a)^p < 0.05 in group of women with I clinical stage compared to group of women with III clinical stage.

^b)^p < 0.05 in group of women with I clinical stage compared to group of women with IV clinical stage.

^c)^p < 0.05 in group of women with II clinical stage compared to group of women with IV clinical stage.

^d)^p < 0.05 in group of women with III clinical stage compared to group of women with IV clinical stage.

^e)^p < 0.05 in group of women with I and II clinical stage compared to control group.

^f)^p < 0.05 in group of women with I, II and IV clinical stage compared to control group.

The mean levels of anti-Hsp60 and anti-Hsp65 antibodies in the patients with ovarian cancer did not differ significantly depending on the cancer histopathological type. In the patients with each histopathological type they also did not differ significantly from the mean levels of these antibodies in the control group. The percentages of positive values for individual histopathological types of ovarian cancer were comparable (details in Table 4).

**Table 4:** Concentrations of anti-Hsp60 and anti-Hsp65 IgG antibodies in group of women with ovarian cancer depending on histopathological type of tumor and in control group

	**Ovarian cancer**			**Controls**
	***Adenocarcinoma papillare serosum***	***Adenocarcinoma mucinosum***	***Adenocarcinoma endometrioides***	**n = 80**
	**n = 82**	**n = 44**	**n = 23**	
**Anti-Hsp60** (AU/ml)	104,17 ± 159,89	82,94 ± 82,87	77,77 ± 83,41	62,42 ± 33,93
(mean ± SD)				
** % of positive results**	26%*	19%	21%	10%
(> 90 percentile for control group)	p = 0.0075	p = 0.1476	p = 0.1535	
**Anti-Hsp65** (AU/ml)	106,41 ± 217,07	78,64 ± 85,73	85,32 ± 92,47	56,35 ± 35,57
(mean ± SD)				
** % of positive results**	21,5%*	15%	29%*	10%
(> 90 percentile for control group)	p = 0.0424	p = 0.3972	p = 0.0200	

*p < 0.05 in group of women with ovarian cancer compared to control group.

Use of chemotherapy as the primary anticancer treatment in ovarian cancer did not resulted in a significant change of anti-Hsp60 antibody levels, which were comparable to levels observed in the group of untreated patients and in the control group. The percentages of positive values in both studied groups of patients were also comparable (Table 5). In the group of patients after chemotherapy the mean anti-Hsp65 antibodies concentration was, however, significantly higher than in the healthy women. The percentages of positive values for anti-Hsp60 levels in the group of untreated patients, and for anti-Hsp65 levels in the group of patients after chemotherapy were also significantly higher than in the group of healthy women.

**Table 5:** Concentrations of anti-Hsp60 and anti-Hsp65 IgG antibodies in group of women with ovarian cancer depending on treatment phase and in control group

	**Phase of antineoplastic treatment**		**Controls**
	**Untreated so far**	**After chemotherapy**	**n = 80**
	**n = 72**	**n = 77**	
**Anti-Hsp60** (AU/ml)	89,59 ± 89,99	99,91 ± 158,40	62,42 ± 33,93
(mean ± SD)			
** % of positive results**	28%*	19%	10%
(> 90 percentile for control group)	p = 0.0041	p = 0.1085	
**Anti-Hsp65** (AU/ml)	80,31 ± 86,71	109,64 ± 226,24	56,35 ± 35,57
(mean ± SD)			
** % of positive results**	19%	22%*	10%
(> 90 percentile for control group)	p = 0.1103	p = 0.0398	

*p < 0.05 in group of women with ovarian cancer compared to control group.

In both studied groups of women – the group with ovarian cancer and the control group of healthy women – concentrations of studied antibodies were not significantly correlated with the age. Levels of anti-Hsp60 and anti-Hsp65 antibodies, however, were positively correlated with each other, both in the group of patients with ovarian cancer and in the control group of healthy women (p = 0.0000, R = 0.35 and p = 0.0000, R = 0.62, respectively).

## Discussion

Ovarian cancer is responsible for as many as 55% of deaths related to malignant genital neoplasms and 6% of all deaths caused by malignant neoplasms in women [11,12]. The prognosis and the long-term survival have remained stable for a long time, mainly due to inadequate diagnostic procedures which usually detect that cancer only at its advanced stage (only 23% of cases are detected at the I stage) [12,13]. Also, a delayed diagnosis is often a consequence of lack of clinical symptoms which sometimes occur only after appearance of local and/or distant metastases [14]. Therefore, a key to significant improvement in treatment results and the prognosis in ovarian cancer is finding methods for early detection of that neoplasm [13]. Expression of CA125 antigen is limited at early stages of ovarian cancer and may also be related to non-malignant lesions; therefore, its prognostic value is only 57% [15]. Determination of that antigen is an example of a method based on detection of circulating tumour-associated antigens – specific proteins released to the circulatory system by neoplastic cells due to their excessive or incorrect expression. Such antigens first have to saturate immunologic antigen-processing capacity and then reach detectable and stable circulating levels, and that occurs only after some time from neoplastic transformation [16]. Excessive or modified expression of specific tumour-associated antigens can also be a source of autoimmunization and antibodies production [17,18]. Presence of antibodies reactive to tumour-associated antigens can be showed in the circulation already at early stages of its development, and much earlier than circulating antigens [19-21]. Furthermore, antibody stability is much higher than other serum biomarkers and less susceptible to effects of various disturbing agents [19,20,22], thus the tumour-reactive antibodies seem to be a more useful diagnostic marker, particularly at early stages of neoplasm development, than tumour-derived antigens [13]. Presence of antibodies against tumour-associated antigens in serum was already demonstrated in patients with various neoplasms [23-25], including ovarian cancer [13,18,26,27]. They were detectable already at early stages of tumour development and related to its progress, as well as allowed distinguishing between benign and malignant lesions (13). However, comparing to other malignant neoplasms, a relatively small number of antigens related to ovarian cancer were found and there is really a small number of studies on antibodies against tumour-associated antigens in ovarian cancer [21]. It seems then that searching for such specific antibodies and their quantitative evaluation may be a key for developing better methods for early diagnosis of that neoplasm.

Recent years have brought many valuable reports on a significant role of heat shock proteins in development of malignant processes, also within the ovary. That role mainly concerns facilitation of malignant transformation, progression of tumour cell survival and contribution to development of resistance to anticancer therapy [1]. However, it is still unknown why Hsps are excessively expressed in tumour cells. Is it caused by an adverse microenvironment of the tumour itself (defensive cellular response) or does it result from genetic modifications related to malignant transformation [28] Neoplastic cells seem to be resistant to pro-apoptotic signals, and as Hsps play an important and comprehensive role in apoptosis processes and at the same time are expressed excessively in malignant cells, they are a subject of intensive research, both as possible therapeutic targets and as prognostic and diagnostic markers [2]. It was proved that excessive expression of various Hsps was related to bad prognosis and poor response to therapy in various types of malignant neoplasms, including ovarian cancer (reviewed in 2). Some Hsps were identified as tumour-associated antigens recognised by antibodies present in serum of patients with ovarian cancer [21], and Hsp27, Hsp70 and Hsp90 expression in tumour tissues was positively correlated to the clinical stage of disease (FIGO) [29]. One of Hsps, which role in malignant neoplastic processes is relatively poorly known, is Hsp60. It seems that in case of prostate cancer increased expression of that protein occurs at an early stage of malignant phenotype development [30], and in rectal and cervical cancers these expression levels increase with malignancy [31,32]. The latest studies showed that in ovarian cancer Hsp60 expression in tumour tissues visibly increased versus expression in correct ovarian tissues [33] and high expression of this protein is also related to poorer prognosis and higher risk of tumour progression [34,35]. Increased levels of anti-Hsp60 antibodies were found in sera of patients with osteosarcomas [36]. The mean concentrations of anti-Hsp60 and anti-Hsp65 antibodies in our group of patients with ovarian cancer were higher than in the control group, but that difference did not reach the statistical significance level. In the group of patients, however, the values considered as positive occurred significantly more often. A very interesting observation was made when the group of women with ovarian cancer was divided depending on the clinical stage of disease (FIGO I – IV). It showed that at the early stages, the mean levels of both studied antibodies were significantly higher than in healthy women and significantly higher than at later stages. The same applies to the occurrence of positive values, which in the group of patients at the I stage occurred in as many as 46% of patients, while in the group of patients at the II stage – in 27% of patients. This observation may point that antigenicity of the tumour changes during neoplastic process or the specific tolerance develops to that antigen, and thus B-cell reactions are weakened. These results indicate usefulness of assessment of anti-Hsp60/65 antibody levels as a diagnostic marker especially at early clinical stages of the disease, when lack of specific markers in serum and lack of clinical symptoms often delay diagnosis. Similar observations were also already made in ovarian cancer for anti-Hsp27 antibodies. In the patients at the I and the II clinical stage of disease the ratio of positive results was 62% and 55%, respectively [37]. Contrary, presence of anti-Hsp90 antibodies is related to later ovarian cancer stages [38]. The mean anti-Hsp60 and anti-Hsp65 antibodies levels did not varied depending on tumour histopathological type, although individual histopathological types differed in positive value ratios.

Recently, a lot is being said about heat shock proteins involvement in development of tumour resistance to non-surgical treatment, and resistance to chemotherapy is one of fundamental problems in treatment of patients with advanced ovarian cancer. One of proteins suspected of participation in development of resistance to chemotherapeutics is Hsp60. Increased expression of this protein was correlated to resistance to cisplatin in various ovarian cancer cell lines [39]. A weak response or even resistance to chemotherapy in ovarian cancer cells also results from increased Hsp27 expression [40]. Hsp60, Hsp27 (and other Hsps) involvement in development of tumour resistance to chemotherapy may result from several mechanisms. As chaperone molecules, they can have cytoprotective effect also on neoplastic transformed cells, “repairing” their proteins damaged by cytotoxic effect of drugs [2] or increasing repair processes in damaged DNA [41,42]. Many authors are of the opinion that the crucial mechanism is, however, protection of tumour cells against apoptosis. The studies suggest this may occur at several stages, through interference with both internal and external apoptosis pathways [4]. Following an analysis of our results it seems that administration of chemotherapy as primary anticancer treatment has no significant effect on anti-Hsp60 antibodies level. An interesting observation concerns, on the other hand, levels of anti-Hsp65 antibodies, which mean value in the group of patients after chemotherapy is significantly higher than in the control group. Anti-Hsp60 and anti-Hsp65 antibodies are extensively described in the literature as cross-reacting antibodies [43,44] due to phylogenetic similarity between forms of these proteins in microorganisms and in mammals. Observations that increased levels of antibodies against mycobacterial Hsp65 (75% homologous with human Hsp60) are related to vascular diseases severity and progress [45,46] resulted in assumptions that immunization against heat shock proteins also affects development and progress of atherosclerosis [47]. As anti-Hsp65 antibodies mediate cytotoxicity against human endothelial cells through cross-reaction with Hsp60 on their surface, damage of vascular cells could result from such reactions in vivo [48]. When levels of anti-Hsp60 and anti-Hsp65 antibodies are assessed simultaneously, usually strong correlation is found between their values [49,50]. In studied by us groups of women that were either healthy or had ovarian cancer, levels of these antibodies were also significantly correlated, although the strength of positive correlation was higher in healthy women (R = 0.62 vs. R = 0.35). Without excluding the cross-reactions mentioned, our results may, however, indicate a diverse nature of both antibodies, e.g., the fact that their cross-reactiveness is only partial. They can recognise different parts of the antigen and have different functional properties. Prohaszka et al. [51] drew similar conclusions from their research, in which they showed differences between anti-Hsp60 and anti-Hsp65 in antigen recognition, complement activation and specificity. Also Handley et al. [52] observed that anti-Hsp60 antibodies present in serum of healthy persons and patients with various autoimmune diseases were competitively inhibited by Hsp60, but only slightly, or not at all, by mycobacterial Hsp65. Research of Metzler et al. [53] showed that antibodies in human serum reacting with human Hsp60 and/or mycobacterial Hsp65 recognised at least three different epitopes in mycobacterial protein. Different functional properties of both antibodies were also proved by research of Birnie et al. [54], who observed that increased levels of anti-Hsp60 antibodies indicated poor prognosis for patients with acute chest pain, while antibodies against mycobacterial Hsp65 had no prognostic value. Significantly higher levels of anti-Hsp65 antibodies in the group of patients with ovarian cancer after chemotherapy, with the mean levels of anti-Hsp60 antibodies comparable to the control group, may also indicate that protein antigenicity was modified by treatment. Possibly post-translational modifications caused in endogenous Hsp60 by chemotherapy, make it homologically more similar to its mycobacterial equivalent, while Hsp60 used in the ELISA test is recombinant protein without these modifications.

There is reactivity and/or cross-reactivity between anti-Hsps antibodies and exogenous Hsps of bacterial origin and endogenous host Hsps, including Hsps circulating in plasma, Hsps present inside cells and on their surface (also neoplastic cells) and Hsps in the extracellular space. These antibodies may control the inflammatory response either positively or negatively, it seems however, they can also have various specific functions in different pathological conditions [7]. Even antibodies against highly homologous Hsps (like human Hsp60 and mycobacterial Hsp65) may be cross-reactive only partially and differ by some functional properties. Detailed knowledge of these differences and properties remains a challenge for the future, particularly considering Hsps and anti-Hsps antibodies involvement in carcinogenesis and neoplasm progression processes, development of metastases and resistance to treatment. Our data indicates that high serum concentrations of anti-Hsp60/65 antibodies are particularly characteristic for early clinical stages of ovarian cancer. However, as they can also be present in healthy persons [55], there is a need to determine the cut-off value and to learn how to distinguish between “normality” and disease using sensitive quantitative techniques [7]. The proposed ELISA technique seems to be such technique. Although diagnostic levels of anti-Hsp60/65 antibodies have not been precisely defined yet, we can assume usefulness of that marker in detection of ovarian cancer, particularly at early clinical stages. The nature of the anti-Hsp immune response in malignant transformation and role of autoantibodies in that process remain to be clarified – is their presence serves as anticancer defence, and if so, whether they can be used as new therapeutic strategies in oncology.

## Competing interests

The authors declare that they have no competing interests.

## Authors’ contributions

PB: author of the concept and principles of work, gathering material, developing the concept and principles of research, laboratory test, description of test results, preparation of literature, co author of the text. RP: author responsible the manuscript, final verification and approval of manuscript, revision and update of literature. AD-B: statistical analysis of results, preparation of the manuscript. All authors read and approved the final manuscript.
